This article has been retracted.

# Design of a Comprehensive Assessment Model for the Stability and Engineering Geology of Slope Based on Improved Convolutional Neural Network

**DOI:** 10.1155/2022/1639311

**Published:** 2022-05-09

**Authors:** Yuedong Liu, Dongdong Yan, Kexiong Zheng

**Affiliations:** No. 3 Geological Brigade of Hebei Geology and Minernal Exploration Bureau, Zhangjiakou, Hebei, China

## Abstract

The geological mechanics, geotechnical characteristics, and hydrogeological conditions of slopes are complex and changeable, so their stability assessment is a complicated system; their traditional engineering geological assessment does not consider the opposition of the system, the uncertainty of performance indicators, and the ambiguity of index classification, being easy to distort results due to the ambiguity. Improved convolutional neural network (CNN) has outstanding advantages in analyzing problems with randomness and fuzziness. It can perform unified numerical processing on slope assessment indicators with precise values, interval values, and qualitative judgment values, making the traditional qualitative description is transformed into quantitative calculation. Therefore, on the basis of summarizing and analyzing previous research works, this paper expounded the research status and significance of the comprehensive assessment model for slope stability and engineering geology; elaborated the development background, current status, and future challenges of the improved CNN; introduced the methods and principles of the model structure, convolutional layer design, and data flow optimization of the improved CNN; performed the assessment index system establishment and index weight determination; established the mathematical assessment model for slope stability; conducted the assessment module design for slope stability based on the improved CNN; analysed the importance of individual factors to the comprehensive engineering geological characteristics; discussed the determination of assessment value of comprehensive unit engineering geological characteristics; explored the assessment module design for slope engineering geology based on the improved CNN; and finally carried out an engineering application and its result analysis. The study results show that the improved CNN can select some universal and objective factors according to the actual conditions of slopes, including topography, stratum lithology, geological structure, atmospheric rainfall, groundwater, engineering activities, setting up factor sets and judgment sets, and making fuzzy inferences. The comprehensive assessment model can use appropriate mathematical methods to judge the pros and cons of slope's stability and engineering geology according to certain principles and standards, and grade the results and identify the most important geological problems. The results of this paper provide a reference for further researches on the design of a comprehensive assessment model for slope stability and engineering geology based on the improved CNN.

## 1. Introduction

Slope stability assessment is an important issue in the construction of open-pit mining, expressway, and water conservancy projects. The assessment results directly affect the way of excavation and support in the early stage of project construction [1]. The slope stability assessment system is a complex system, and its physical and mechanical properties and hydrogeological conditions are complex and changeable. As far as the current engineering geological exploration methods and technical means are concerned, it is still difficult to accurately judge the stability state and other engineering geological conditions before construction [2]. Comprehensive assessment of engineering geology refers to the evaluation of its pros and cons by selecting appropriate mathematical methods in accordance with certain principles and standards on the basis of the investigation of the engineering geological environment and classifying the assessment results to determine the existence of process systems for the most important geological problems [3]. Since the slope stability analysis belongs to dynamic system engineering, which is of guiding significance for the construction of slope engineering. Slope engineering geology does not consider the opposition of the system, the uncertainty of the assessment index and the ambiguity of the index classification, which is easy to make the assessment results. Commonly used assessment methods include comprehensive index method, analytic hierarchy process, and fuzzy comprehensive assessment method, and each method has its own characteristics, but there are certain limitations when using it [4].

The outstanding performance of convolutional neural network (CNN) in fields such as machine-learning and computer vision has led to its application in the solution of more problems. The advantage of CNN is that it can automatically extract features, so as to avoid the difficulty and trouble of manual feature extraction. For classification tasks, the problem of overfitting is reflected in a low error rate on the training set and a high error rate on the test set [5]. Overlearning takes the special characteristics of a certain type of data in the training set as the general characteristics of this type of data, so that when the learned model is tested on the test set data, the special characteristics of this type of data are judged as general characteristics, and data cannot be accurately classified with a high error rate [6]. This is a ubiquitous and rather intractable problem in supervised learning, and therefore needs to be improved on the overfitting problem of CNN. In order to further improve the generalization ability of the model, the optimized model can improve the performance of the neural network structure through dropout [7]. Randomly ignoring the neurons in the convolutional layer can train a large number of different network structures in a reasonable time, while reducing the interaction between neurons in the hidden layer and optimizing the structure of the model [8]. The improvement of the convolution layer is mainly divided into the method of using parallel and series sharing of the network for larger convolutions and the method of directly using parallel connection for smaller convolutions. The improvement of the model mainly is the convolutional and fully connected layers that consume a lot of parameters and training time.

This paper will expound the research status and significance of the comprehensive assessment model for slope stability and engineering geology; elaborate the development background, current status, and future challenges of the improved CNN; introduce the methods and principles of the model structure, convolutional layer design, and data flow optimization of the improved CNN; perform the assessment index system establishment and index weight determination; establish the mathematical assessment model for slope stability; conduct the assessment module design for slope stability based on the improved CNN; analyse the importance of individual factors to the comprehensive engineering geological characteristics; discuss the determination of assessment value of comprehensive unit engineering geological characteristics; explore the assessment module design for slope engineering geology based on the improved CNN; and finally carry out an engineering application and its result analysis. The detailed chapters are arranged as follows: Section 2 introduces the methods and principles of the model structure, convolutional layer design, and data flow optimization of the improved CNN; Section 3 conducts the assessment module design for slope stability based on the improved CNN; Section 4 explores the assessment module design for slope engineering geology based on the improved CNN; Section 5 carries out an engineering application and its result analysis; and Section 6 is conclusion.

## 2. Methods and Principles

### 2.1. Model Structure for Improved CNN

The improved CNN model structure can carry out unified numerical processing for slope assessment indexes with exact value, interval value, and qualitative language judgment value. For a convolutional layer, assuming that it has *n* convolution kernels of size *a*^*∗*^*b*^*∗*^*c*, it performs convolution processing on images of size *a*_1_^*∗*^*b*_1_^*∗*^*c*_1_, the stride is *i*, and the number of zero-padded layers is *d*, then the feature map size *A*_*i*_ generated after convolution is as follows:

(1) $$\begin{array}{c} A_{i}=\sum_{i=1}^{n}\left(\frac{a_{i}+b_{i}+c_{i}}{d}-\frac{a_{1i}+b_{1i}+c_{1i}}{d}\right)=\sum_{i=1}^{n}\frac{f_{i}}{e_{i}}\cdot \frac{B_{i}+C_{i}+D_{i}}{d\cdot E_{i}}, \end{array}$$

where *B*_*i*_ and *C*_*i*_ are the expectation and variance of each batch of input data; *D*_*i*_ is the output of the *i*th convolutional layer; *E*_*i*_ is the weight matrix of the *i*th fully connected layer, *E*_*i*_ is the bias of *D*_*i*_; *f*_*i*_ is the predicted value; and *e*_*i*_ is the actual label value.

The optimization method adopts the stochastic gradient descent algorithm to optimize the objective function. According to the operation rules of the gradient descent method, it needs to find the gradient of the weight to the cost function to update the weight, and then the update rule *F*_*i*_ of the weight of the *i*th layer can be expressed as follows:

(2) $$\begin{array}{c} F_{i}=\sum_{i=1}^{n}\frac{g_{i}}{g_{i-1}}-\frac{h_{i}}{g_{i}}=\sum_{i=1}^{n}\frac{l}{k}\cdot \frac{g_{i}}{h_{i}}, \end{array}$$

where *g*_*i*_ is the error coefficient of the *i*th layer, which indicates the degree of responsibility of the layer's error to the total error; *g*_*i*−1_ is the output of the *i*−1 layer, which is the input of the first layer; *h*_*i*_ is the output of last fully connected layer and is usually a feature vector; *l* is the index in the feature vector; and *k* is the output feature value processed by the activation function.

The first-level fuzzy assessment only reflects the influence of each single factor on the main object of the first-level assessment; the fuzzy comprehensive assessment considers the influence of all factors, and the final assessment result can be expressed as follows:

(3) $$\begin{array}{c} G_{i}=\sum_{i=1}^{n}m_{i}\left|\frac{o_{i}}{\sum_{i}^{n}1/p_{i}}\right|, \end{array}$$

where *G*_*i*_ is the fuzzy relationship between the universe of discourse *F*_*i*_ and the assessment set *A*_*i*_; *m*_*i*_ is the hierarchical fuzzy vector; *o*_*i*_ is the weight set; *p*_*i*_(*i* = 1, 2,..., *n*) is the fuzzy comprehensive assessment index according to the maximum membership degree principles.

Usually a CNN is represented as a series of layers that form a directed acyclic graph model, and the connections of these layers are done through a high-level description scheme. Therefore, it maps the directed acyclic graph model to the hardware model, that is, the synchronous data flow model, which is similar to building blocks to instantiate each layer into a module and then connect to each other. The computing process realizes uninterrupted pipeline operation, and the node operation method of input and output improves the robustness of the system to a certain extent because the design of each layer drives data flow independently, thus forming a heterogeneous flow mode [9]. In this input-output mode, the output data flows out immediately instead of being buffered on on-chip memory, saving the memory usage of the entire network. The model trains the CNN offline to obtain model files of weights and bias parameters, and designs a fixed-point quantization algorithm. According to the chain rule and the principle of back propagation, the input, output, and accurate value are compared and evaluated in the form of loss function, so as to adjust the parameters such as weight and bias. The assessment model is trained using a calibrated data set, and the weights and bias parameters of the CNN model are obtained from offline pretraining.

### 2.2. Convolutional Layer Design and Data Flow Optimization

For the coordinate position, the convolutional layer will set a unique vector for identification. Specifically, for each position, concatenating the data flow vector *q*_*i*_ can deduce the position vectors *q*_*i*1_ and *q*_*i*2_ of the two entities; depending on the direction vector *r*_*i*_ and the dependent feature vector *s*_*i*_, and the representation vector *H*_*i*_ of the data flow can be obtained as follows:

(4) $$\begin{array}{c} H_{i}\left(x\right)=\sum_{i=1}^{n}\frac{v\left(x\right)}{u}\cdot \frac{q_{i}}{r_{i}+s_{i}}=\sum_{i=1}^{n}\frac{y_{i}}{w}\cdot \frac{q_{i}}{r_{i}+s_{i}}, \end{array}$$

where *u* is the bias term; *v*(*x*) is a nonlinear function; *w* is the number of convolution kernels; and *y*_*i*_ is the probability that there is a relationship between entities *q*_*i*1_ and *q*_*i*2_ at this position.

The development degree of engineering geological structure plane, slope height, slope inclination, and so on belong to the smaller the better index, so the relative membership degree of the index and the relative membership degree of the level can be given the initial weight vector *J* = {*j*_1_, *j*_2_,…, *j*_*n*_} and normalize the vector *J* to obtain the weight vector:

(5) $$\begin{array}{c} J_{i}\left(x\right)=\left\{\frac{I\left(x\right)}{\sum_{i}^{n}j_{i}},\frac{K\left(x\right)}{\sum_{i}^{n}j_{i}},\frac{L\left(x\right)}{\sum_{i}^{n}j_{i}},\frac{M\left(x\right)}{\sum_{i}^{n}j_{i}},\frac{N\left(x\right)}{\sum_{i}^{n}j_{i}}\right\}, \end{array}$$

where *I*(*x*) is the damping factor; *K*(*x*) is the unit matrix; *L*(*x*) is the hierarchical fuzzy vector; *M*(*x*) is the weight set of the fuzzy relationship; *N*(*x*) is the fuzzy comprehensive assessment index and determines its rank according to the maximum membership principle.

The comprehensive engineering geological assessment *O*_*i*_(*x*) of the unit is carried out on the basis of the assessment of each individual factor, which is related to the nature and importance of each individual factor. The specific calculation formula is as follows:

(6) $$\begin{array}{c} O_{i}\left(x\right)=\sum_{i=1}^{n}\frac{P_{i}\left(x\right)-Q_{i}\left(x\right)}{R_{i}\left(x\right)}, \end{array}$$

where *P*_*i*_(*x*) is the proportional factor between the value weight and the importance of the influence weight; *Q*_*i*_(*x*) is the influence of all other factors on the factor *i*; *R*_*i*_(*x*) not only shows the influence of a certain factor on the geological characteristics, also reflects the mutual influence of various factors and the optimization and rationality of each factor in engineering geological assessment.

From the perspective of the whole process, the CNN is equivalent to a function. Given specific file information, the output value is a feature value representing the file, and the feature value can be used to represent the user's rating on the item text assessment information. In order to further improve the generalization ability of the model and prevent overfitting, optimizing the model can improve the performance of the neural network structure through dropout. Dropout means that in training, some neurons in the hidden layer work, and some neurons do not work. Randomly ignoring the neurons in the convolutional layer can train a large number of different network structures in a reasonable time, while reducing the interaction between neurons in the hidden layer and optimizing the structure of the model [10]. The improved CNN model can determine how many feature extractors by setting the number of convolution kernel filters in the network initialization. The cross-channel model uses multiple variable-length convolution kernel filters to obtain more feature information and add a layer of cross-channel convolution kernel behind linear convolution filter to achieve cross-channel. When the number of iterations is the same, the cyclic learning rate strategy obviously has higher recognition accuracy, that is, when the same accuracy is achieved, the cyclic learning rate strategy obviously requires less iteration.

## 3. Slope Stability Assessment Based on Improved CNN

### 3.1. Establishment of Assessment Index System and Determination of Index Weight

For a given assessment area, there are many factors affecting the comprehensive engineering geology of the slope, mainly including the bearing capacity of rock upper body, groundwater level, groundwater chemical composition, topographic relief, environmental changes, earthquakes, denudation, and artificial activities. Specific geological bodies have their own unique influencing factors, which require the model to comprehensively consider all factors in the comprehensive engineering geological assessment of slopes, that is, comprehensive analysis and assessment of engineering geological conditions, social benefits, and economic benefits. It is not difficult to imagine that each influencing factor has different effects on the slope due to the difference in different units; the optimal factor relative to one unit may be a general factor in another unit. Therefore, the properties of a single factor are not only related to the best and worst values of the factor in the entire slope, but also related to the representative value of the factor in the unit where it is located. As far as the relationship between various factors is concerned, the change of a certain factor will cause the change of other factors. An assessment without considering the interaction between factors will be a partial-coverage conclusion. Therefore, the assessment of the engineering geological characteristics of slope must adopt a comprehensive method and consider it comprehensively, in order to obtain more accurate data for the assessment of the slope stability [11].  Figure 1 shows framework for the establishment of assessment index system and the determination of index weight in slope stability assessment based on the improved CNN.

The expert survey method is based on the experience of experts to give the weight of each factor, and the assessment results are highly subjective; the entropy method is to determine the weight by mathematical methods based on the relationship between the original data, which is very objective, but sometimes the obtained weights are inconsistent with the real situation. The improved CNN performs unified numerical processing on the slope assessment indicators with precise values, interval values and qualitative language judgment values, so that the traditional qualitative description is transformed into quantitative calculation. The improvement of the model mainly improves the convolutional and fully connected layers that consume a lot of parameters and training time. The improvement of the convolution layer is mainly divided into the method of using parallel and series sharing of the network for larger convolutions and the method of directly using parallel connection for smaller convolutions. Since the fully connected layer occupies a large number of parameters, it is easy to cause overfitting to replace all the fully connected layers. This paper mainly improves the convolutional layers and fully connected layers that occupy more parameters in the original CNN. Replacing the fully connected layer with a scale normalization layer can reduce a lot of time and the efficiency of the algorithm is improved, so that the entire network structure achieves the purpose of reducing the training time and improving the accuracy.

In order to highlight the risk indicators in the assessment, the model uses the penalty local variable weight principle to construct a local state variable weight function, that is, penalizes the difference of the indicators, and neither punishes nor encourages the good value of the indicators. The variable weight assessment avoids the index neutralization phenomenon that occurs in the constant weight assessment, and the assessment results better reflect the outstanding impact of unfavourable geological environmental conditions on the development and construction of the pipe gallery [12]. The distribution of partitions in the variable weight assessment partition map is more compact and concentrated, which is convenient for partition division. By adjusting the weight of the risk index, the punishment of the risk index is realized, and the influence of unfavourable geological environment conditions on the suitability assessment is highlighted. Given a very small initial value of the learning rate based on experience, the learning rate is linearly increased on the initial basis at a very low rate that is not the initial learning rate, and the loss value is plotted against the learning rate. The learning rate range corresponding to the region where the loss value decreases the fastest is the cyclic variation range of the optimal learning rate, and the upper and lower bounds of the range are called the maximum boundary and the minimum boundary.

### 3.2. Establishment of Mathematical Assessment Model for Slope Stability

Under the influence of various natural and man-made factors, the slope has been constantly developing and changing, restricted by factors such as time and space. These factors have obvious ambiguity and uncertainty, and it is difficult to express with exact numbers. It not only combines the advantages of the qualitative analysis of the expert survey method but also selects an appropriate mathematical model for quantitative analysis, which is suitable for determining the weights of factors affecting slope stability. Normative unification can eliminate the influence of qualitative judgment of assessment indicators and the subjective arbitrariness of expert authoritative assessment and better consider the interaction and effect of various qualitative and quantitative assessment indicators (Figure 2). When evaluating slope stability using the improved CNN method, disaster factors with certain universality and objective reality should be selected according to their formation conditions, including topography, stratum lithology, geological structure, atmospheric rainfall, groundwater, engineering activities, and other factors, so as to establish a factor set and a judgment set and make fuzzy inferences. The random pooling method randomly selects the pooling activation value at the pooling layer during training, and then applies the probability of each unit in pooled region as the model average of the weighted probability during testing.

The slope rock formation tendency is the same as that of the side slope, and the layer controls the failure surface of the slope. There are more than two groups of tectonic joints developed in the bedding slopes in the study area, and there are many weak planes in the inter-layer. When the inclination angle of the rock layer is greater than the slope angle, the weak structural plane has no free surface in the inclination direction, and the rock layer generally does not cause the slope to slip and fail but is prone to dumping damage [13]. As shown in Figure 3, the rock mass begins to bend as a cantilever beam in the direction of the air at the front edge, and gradually develops into the slope, causing the rear edge of the slope to crack, forming reverse slope steps and grooves parallel to the strike. The determination of factor membership degree adopts the expert assessment method and the formula method. The expert assessment method is mainly used to obtain the value, and for continuous variables, a membership function representing the relationship between membership degree and index value is established. When the shear stress of the fracture zone in the slope exceeds its shear strength, the slope gradually dislocates and slides down to form a collapsed sliding mass. This type of slope belongs to a relatively stable structure type and does not have the basic geological conditions for deformation and damage.

The comprehensive assessment model of slope stability and engineering geology is a typical complex system problem. The uncertainty analysis method of variable fuzzy sets based on relative difference has obvious advantages, but the construction process of variable fuzzy sets is complicated. This paper discusses the application of set-pair analysis fuzzy connection degree between samples and grades to construct variable fuzzy sets to improve the reliability and versatility of quantitative analysis. The size of the weight reflects the relative position of each factor in the assessment of the suitability of construction land, and the larger the weight, the greater the effect of the factor. The factors involved can be determined by corresponding subjective and objective methods according to the characteristics of the geological environment of the assessment unit [14]. The determination of the membership degree of the assessment index is the key of fuzzy comprehensive assessment. When the sliding force of the body is greater than the anti-sliding force on the sliding surface, the rock mass of the slope slides along the underlying weak face in the direction of the front of the slope, and the sliding body pulls the disintegrating body. When the lower part of the slope is blocked from sliding, bending deformation occurs until the penetration failure.

## 4. Slope Engineering Geology Assessment Based on Improved CNN

### 4.1. Individual Factors of Comprehensive Characteristics of Engineering Geology

The comprehensive assessment model of engineering geology should start with the study of the deformation and failure mechanism of the slope. Under the premise of avoiding the overlapping of factors among the indicators, the geological conditions of the slope should be comprehensively considered, and the factors that have a greater impact on the deformation and failure of the slope should be selected as assessment indicators. The individual factors realize uninterrupted pipeline operation and improve the robustness of the system to a certain extent because the design of each layer drives data flow independently. General geological conditions include geological structure characteristics, topographic, and geo-morphological characteristics, hydrogeological characteristics, and deformation and failure characteristics of slopes (Figure 4). Geological structural features include rock and soil type, structural surface features, physical and mechanical properties of rock and soil structure; topographical features include bank slope height, slope, development degree of gullies, and so on.; hydrogeological features include water surface width, wind and wave action, groundwater, and so on. Based on the plane coordinate grid, the divided rectangle is used as the assessment unit, and the size of the unit can be determined according to the actual situation. The indicators that reflect the assessment plan often have different dimensions and orders of magnitude, and it is necessary to normalize all indicators, that is, to uniformly transform the attribute values of the assessment indicators into a certain range and have the same impact trend [15].

The weights of assessment indicators are determined by combining expert scoring. Each expert independently compares the relative importance of the factors in each layer to the objectives of the previous layer, constructs a judgment matrix, and then collects the judgment matrix constructed by each member to obtain a comprehensive judgment matrix. After discussion and revision by all experts, all experts have no opinion on the comprehensive judgment matrix, then the corresponding eigenvector are calculated, and the consistency test of judgment matrix is carried out [16]. On the basis of analyzing the geological background of the slope and the main geological environmental problems, the comprehensive assessment index system of the slope geological environment is constructed, which includes the element layer, the index layer, and the variable layer. The element layer has four elements: geological background factor, geological disaster factor, environmental pollution factor, and resource destruction factor.  Table 1 shows an example of trained results of improved CNN by convolutional layer design and data flow optimization. The index layer consists of 16 indicators: rock type, fault density, vegetation coverage, catchment area, joint development degree, relative height difference, ground collapse, collapsed slope, karst collapse, water environment pollution, soil pollution, biological chain pollution, destruction of vegetation, destruction of topography and landscape, destruction of water environment and water resources, and destruction of land resources.

The convolution layer performs convolution calculation on the two-dimensional data through the convolution kernel and adds the bias vector to obtain the feature map of the initial feature extraction and uses the weighted summation of multiple feature maps as the input of the subsampling layer, so as to obtain the nonlinear feature map. New feature maps for linear feature grabbing. The core of the improvement is to use a locally optimal sparse structure to replace the original full connection method and use a multilayer to replace the traditional method of adding a large number of filters to the traditional convolution layer, to avoid redundancy to the greatest extent, and to use dense computing to achieve the acceleration of training process. The basic idea of the multifactor and multilevel model is to divide many factors into several levels, first make a comprehensive assessment of each factor at the lowest level, and then make a comprehensive assessment of each factor at the upper level and proceed to the highest level to obtain the overall assessment result. Adding redundant classifiers to the underlying structure allows the underlying trainable parameters to be more fully trained during gradient descent. The principle is that it has a normalization effect to a certain extent, so adding a batch normalization processing structure or a dropout processing structure before the classifier will play a greater role. At the same time, redundant classifiers really play a role after the network structure approaches convergence, and isolation measures are adopted in the early stage of training, which can save computing resources.

### 4.2. Assessment Value of Comprehensive Characteristics of Engineering Geology

Since different types of projects have different requirements for foundation quality, the weights are adjusted according to the geological environment, geotechnical properties of the comprehensive assessment model of engineering geology, and the degree of influence of the spatial distribution of soft soil on different types of projects. The assessment value of comprehensive characteristics of engineering geology can train a large number of different network structures in a reasonable time, while reducing the interaction between neurons in the hidden layer and optimizing the structure of the model. By synthesizing the overall influence of various factors on various projects, the model assigns weights to the degree of influence of various factors on engineering diseases to evaluate and draws a comprehensive zoning assessment map of engineering geology based on the assessment results [17]. As shown in Figure 5, the improved CNN model has the advantages of both single-layer neural network and multilayer neural network. In the case of less training data, the model can still obtain excellent training parameters through interlayer transfer in image feature extraction, so it builds a feature model. If the input is further away from the parameter vector, the output of the radial basis function will be larger. It can be understood in this way that the output of the radial basis function is a penalty term that weighs the matching degree of a model of the class associated with the radial basis function.

The comprehensive assessment model of slope stability and engineering geology based on improved CNN needs to include three conditions of geology, environment, and engineering. Among them, geological conditions include compressive strength, elastic modulus, Poisson's ratio, cohesion and internal friction angle; environmental conditions involve maximum process rainfall, underground water seepage; engineering conditions include slope height, slope gradient, seismic intensity, and explosive particle vibration velocity. Slope stability will be divided into 5 grades: extremely stable, stable, basically stable, unstable, and extremely unstable. The improved CNN has outstanding advantages in analyzing problems with randomness and fuzziness. Since the slope stability analysis belongs to dynamic system engineering, the slope stability is affected by many factors, and the cloud model is applied to the slope stability. In the qualitative assessment, the reliability of the assessment results can be guaranteed, and a new idea of quantitative analysis is provided for the assessment of qualitative concepts. The size of the convolution kernel is the feature size of the upper layer, and the result after convolution is a node, which corresponds to a point in the fully connected layer. The feature map loses its spatial topology in the fully connected layer, is expanded into a vector and passed to the next layer through the excitation function [18].

## 5. Engineering Application and Result Analysis

### 5.1. Experimental Platform and Project Overview

The experimental operating system is Windows 10 64-bit operating system, and the graphics card is NVIDIA GeForce GTX 760. The experiment in this paper uses Google's open-source deep-learning framework Tensorflow and uses CUDA acceleration. In order to judge the effectiveness of the proposed improved method, a total of 3 control groups were set up in the experiment: the first group improved the LeNet5 model and tested it with the Cifar10 data set; the second group input Cifar10 data of different sizes to test the improved model testing; the third group refines the Alexnet model. The assessment index of the experiment is 4 items: the change curve of loss function, the change curve of accuracy rate, the consumption time, and the amount of model parameters, among which the change curve is generated after fitting the experimental data. The improved model must ensure that the loss function has decreased enough, the accuracy rate cannot be lower than before the improvement, the time required for training is basically the same or reduced, and the number of parameters required by the model has decreased compared with that before the improvement. Examples of experimental platform simulation stable and unstable slope are given in Figure 6.

The superficial layer of the slope area is relatively loose collapsing rubble soil, and below it is the ancient slope deposit, and the clay content in the deposit is relatively high, and the clay soil at the front edge of the slope body is in a soft plastic state. The comprehensive assessment model considers the value of the shear strength of the potential sliding surface of the deformed slope. The sliding-band gravel soil exposed by the borehole needs to be subjected to shear strength tests under different moisture contents. The analysis of the influence of water on the shear strength parameters of the sliding zone soil influences the error of the empirical method in the value of the shear strength parameters of the crushed soil. When evaluating the stability of a deformed slope, there are many assessment factors, and each factor plays a different role in the assessment [19]. According to the deformation failure characteristics, formation mechanism analysis and stability assessment results of the deformed slope, the model will give corresponding suggestions for treatment measures. In view of the deformation and failure characteristics of deformed slopes, the idea of zoning treatment is adopted for reinforcement, which is using frame anchor cables or antisliding piles to strengthen the slope body in zones, and finally strengthen the foundation of penstock pipe piers to achieve governance. As there are many factors that affect the deformation of the slope, and there are intricate connections between the factors, the stability assessment of the deformed slope needs to be evaluated according to the specific situation.

### 5.2. Result Analysis

This kind of network will more or less have problems such as information loss and gradient easily disappearing during the training process. The residual module can alleviate the ability of gradient vanishing to a certain extent, and it is added to the CNN model, and an improved CNN is proposed. In order to prevent multiple neurons in the network from learning the same content and improve the training effect, before network training. As there is no uniform standard for the selection of parameters in the network, and the network models constructed based on different data sets will have different training effects on the selection of different network parameters, it is necessary to select a suitable network according to the comparison and analysis of the actual data set [20]. Active local reduction of rock strata combination is suitable for when the number of layers is small, various rock stratum combination reduction calculations can be performed, and the obtained results can reflect the slope deformation controlled by different rock layers on the entire slope different forms of destruction (Figure 7). When the strength is reduced, the instability of the slope is often controlled by the strength reduction of the local rock and soil mass, which is very obvious in the heterogeneous slope. Therefore, in the reduction process, only the strength of local rock and soil elements is reduced, and the parameters of other rock and soil elements remain unchanged.

The improved CNN model has the advantages of both single-layer neural network and multilayer neural network, so compared with previous research, this comprehensive assessment model for the slope stability and engineering geology is to use a locally optimal sparse structure to replace the original full connection method, and use a multilayer to replace the traditional method of adding a large number of filters to the traditional convolution layer, to avoid redundancy to the greatest extent, and to use dense computing to achieve the acceleration of training process. In recent years, with the development of computer technology and modern applied mathematical theory, nonlinear mathematical theory has been widely used in comprehensive assessment of engineering geology such as slope stability due to its advantages in comprehensive decision-making. The comprehensive assessment process of engineering geological environment mainly includes the construction of assessment index system and quantitative classification, determination of index weights, establishment of mathematical assessment models, division of assessment units, comments on assessment results, and drawing of assessment maps. The complexity of the engineering geological environment determines that its assessment must be carried out using the theory of complex large systems and the method of comprehensive integration, that is, through the principle of decomposition and coordination, quantitative analysis is carried out under qualitative analysis [21]. This method can overcome the drawbacks of the unique solution in the traditional mathematical method, and obtain multiple levels of problem solutions according to different possibilities, which is scalable in the assessment model for slope engineering geology.

The feature of structural plane is an important factor affecting the stability of rock, and the spacing of structural plane can reflect the influence degree of geological structure on rock mass. To simplify the calculation, the roughness, continuity, weathering, and cementation degree of structural plane are integrated into structural plane feature. Clay rock swells and shrinks when it encounters water, and its strength is greatly affected by groundwater, but the clay rock stratum has poor water permeability and no obvious groundwater was seen during the construction process. The main algorithm idea of the improved CNN algorithm is to first calculate the distance between the data to be classified and the known classified data, find the sample with the closest distance to the sample to be classified and then discriminate the data to be classified according to the category to which the classified sample belongs [22]. If the most adjacent samples of the sample data to be classified all belong to a category, then the sample to be classified also belongs to this category; otherwise, the category with the majority is used to determine which category the sample to be classified belongs to. The comprehensive assessment model of engineering geology first uses a multilayer CNN to preclassify the data, and then uses the output of the preclassification process as the input of the improved algorithm and uses the improved algorithm to make classification decisions.

## 6. Conclusion

This paper performed the assessment index system establishment and index weight determination, established the mathematical assessment model for slope stability, conducted the assessment module design for slope stability based on the improved CNN, analysed the importance of individual factors to the comprehensive engineering geological characteristics, discussed the determination of assessment value of comprehensive unit engineering geological characteristics, explored the assessment module design for slope engineering geology based on the improved CNN and finally carried out an engineering application and its result analysis. Fuzzy comprehensive assessment method is widely used in multilevel, multifactor, and multi-index comprehensive assessment of environmental quality, especially in the comprehensive assessment of engineering geology. The determination of the membership degree of the assessment index is the key of fuzzy comprehensive assessment. When the sliding force of the body is greater than the antisliding force on the sliding surface, the rock mass of the slope slides along the underlying weak face in the direction of the front of the slope, and the sliding body pulls the disintegrating body. This method can overcome the drawbacks of the unique solution in the traditional mathematical method and obtain multilevel problem solutions according to different possibilities. The principle of the improved neural network has a normalization effect to a certain extent, so adding a batch normalization processing structure or a dropout processing structure before the classifier will play a greater role. The study results show that the improved CNN can select some universal and objective factors according to the actual conditions of slopes, including topography, stratum lithology, geological structure, atmospheric rainfall, groundwater, engineering activities, setting up factor sets and judgment sets, and making fuzzy inferences. The comprehensive assessment model can use appropriate mathematical methods to judge the pros and cons of slope's stability and engineering geology according to certain principles and standards and grade the results and identify the most important geological problems. The results of this paper provide a reference for further research on the design of a comprehensive assessment model for slope stability and engineering geology based on the improved CNN.

## Figures and Tables

**Figure 1:** Framework for the establishment of assessment index system and the determination of index weight in slope stability assessment based on improved CNN.

**Figure 2:** Establishment of mathematical assessment model for slope stability based on improved CNN.

**Figure 3:** Model structure for improved CNN and its convolutional layer design and data flow optimization.

**Figure 4:** Example of rose diagrams of geological structure strikes of a stable slope (a) and an unstable slope (b).

**Figure 5:** Assessment value for comprehensive characteristics of engineering geology of a stable slope (a) and an unstable slope (b).

**Figure 6:** Example of experimental platform simulation stable (a) and unstable (b) slope.

**Figure 7:** Relationship between predicted bias rate and iteration in the assessment model for the stability and engineering geology of slope based on improved CNN.

**Table 1:** Example of trained results of improved CNN by convolutional layer design and data flow optimization.

Sample	Expected output				Trained output		Accuracy
1	0.04	0.01	0.06	0.000283	0.000644	0.000114	0.999940
2	0.03	0.02	0.01	0.000473	0.000376	0.000333	0.994860
3	0.05	0.08	0.05	0.000123	0.000225	0.000603	0.996368
4	0.02	0.03	0.03	0.000765	0.000996	0.000267	0.999086
5	0.01	0.07	0.09	0.000836	0.000301	0.000746	0.998954
6	0.03	0.05	0.04	0.000538	0.000788	0.000346	0.998648
7	0.09	0.05	0.07	0.000853	0.000656	0.000295	0.991684
8	0.03	0.02	0.04	0.000327	0.000093	0.000030	0.990463
9	0.01	0.05	0.06	0.000838	0.000139	0.000428	0.995258
10	0.06	0.03	0.02	0.000264	0.000773	0.000463	0.996486

## Data Availability

The data used to support the findings of this study are available from the corresponding author upon request.
